The article "Skin boosters: Definitions and varied classifications" was retracted in 2025. Reasons: plagiarized images; overlap with other authors' work; compromised peer review; concerns about the images.

# Skin boosters: Definitions and varied classifications

**DOI:** 10.1111/srt.13627

**Published:** 2024-03-13

**Authors:** Kyu‐Ho Yi, Waranaree Winayanuwattikun, Sung‐Yeon Kim, Jovian Wan, Vanravi Vachatimanont, Ardhiah Iswanda Putri, Inneke Jane Hidajat, Yuri Yogya, Ruri Pamela

**Affiliations:** ^1^ Division in Anatomy and Developmental Biology Department of Oral Biology Human Identification Research Institute BK21 FOUR Project Yonsei University College of Dentistry Seoul South Korea; ^2^ Maylin Clinic (Apgujeong) Seoul South Korea; ^3^ Division of Dermatology Faculty of Medicine Ramathibodi Hospital Mahidol University Bangkok Thailand; ^4^ VS Line Clinic Incheon South Korea; ^5^ Asia‐Pacific Aesthetic Academy Honk Kong Hong Kong; ^6^ iSKY Center Bangkok Thailand; ^7^ Rejuva Clinic Surabaya Indonesia; ^8^ Department of Dermatology Faculty of Medicine Atma Jaya Catholic University of Indonesia Jakarta Indonesia; ^9^ Department of Dermatology and Venereology Universitas Padjadjaran Bandung Indonesia; ^10^ CELV Dermatology Clinic Jakarta Indonesia

**Keywords:** botulinum neurotoxin, exosome, growth factor, hyaluronic acid filler, polydeoxyribonucleotide, poly‐D‐lactic acid, poly‐L‐lactic acid, polynucleotides, secretome, skin booster

## Abstract

**Background:**

The concept of “skin boosters” has evolved, marking a shift from traditional uses of hyaluronic acid (HA) fillers primarily for augmenting skin volume to a more diverse application aimed at improving dermal conditions. Restylane Vital and other HA fillers have been repurposed to combat skin aging and wrinkles by delivering HA directly to the dermis.

**Objectives:**

This review aims to define the term “skin booster” and to discuss the various components that constitute skin boosters. It seeks to provide a comprehensive overview of the different ingredients used in skin boosters, their roles, and their impact on enhancing dermal conditions.

**Methods:**

A comprehensive review was conducted, focusing on representative skin booster ingredients. The approach involved analyzing the different elements used in skin boosters and their specific roles in enhancing dermal improvement.

**Results:**

The findings indicate that skin boosters, encompassing a range of ingredients, are effective in improving the condition of the skin's dermis. The review identifies key ingredients in skin boosters and their specific benefits, including hydration, elasticity improvement, and wrinkle reduction.

**Conclusions:**

Skin boosters represent a significant development in dermatological treatments, offering diverse benefits beyond traditional HA fillers. This review provides valuable insights into the constituents of skin boosters and their effectiveness, aiding readers in making informed decisions about these treatments. The potential of skin boosters in dermatological practice is considerable, warranting further research and application.

## 1 INTRODUCTION

The phrase “skin booster” has gained prominence within the esthetic industry, denoting the application of hyaluronic acid (HA) filler products with low cross‐linking to deliver HA into the skin's dermal layer, aiming to improve skin aging and diminish wrinkles. While HA fillers were initially utilized primarily for augmenting volume, the use of these fillers in skin boosting emerged to enhance skin condition by fortifying the extracellular matrix (ECM) in the dermal layer. Although trademarks such as Restylane Skinboosters “Vital” and “Vital Light” exist, the term “skin‐booster” has evolved into a widely used generic descriptor, akin to the way “Botox” is universally employed to refer to botulinum toxin (BoNT) products in procedures conducted by Allergan.

Skin boosters contribute significantly to decelerating and ameliorating the skin aging process. The aging of the skin involves a decline in the quantity of epidermal and dermal cells, the diminishment of rete ridges, reduced levels of collagen and elastin, and a decrease in glycosaminoglycans. Additionally, heightened levels of reactive oxygen species contribute to the breakdown of antioxidants in tissues, resulting in a diminished antioxidant effect, activation of melanocytes leading to skin darkening, and an increase in pigmentation irregularities. Skin boosters intervene in these processes by enhancing and fortifying the extracellular environment, ameliorating pigmentation issues, inflammation, and vasodilation to manifest their beneficial effects.

While there exists an increasing diversity in the types and objectives of skin boosters within the realm of esthetic practices, a specific, comprehensive definition for this term has not yet been established. Nevertheless, it is logical to consider defining skin boosters as encompassing a wide array of ingredients employed to enhance and improve skin condition.

## 2 CLASSIFICATION OF SKIN BOOSTERS

### 2.1 Hyaluronic acid

Fillers with diverse characteristics, including variations in filler particle size, reduced cross‐linking, and enhanced injection comfort, have been developed by numerous companies and widely employed in commercial applications. HA is naturally found in the dermal layer of the skin, renowned for its capacity to retain moisture, support hydration, and stimulate the secretion of growth factors (GFs) within the skin's connective tissues.^1^

The randomized clinical trial of Gao et al.,^2^ involving 129 females with varying ages and skin types examined the effects of orally administered HA on skin health. The study revealed significant improvements in skin hydration within 2–8 weeks for both young and elderly participants, followed by enhanced skin tone after 4–8 weeks and increased epidermal thickness after 12 weeks of HA intake. Overall, the findings strongly support the efficacy of oral HA supplementation in promoting skin health across diverse age groups and skin types.

In the context of HA skin boosters, two types can be distinguished: non‐cross‐linked and low‐cross‐linked HA. HA skin boosters serve various purposes such as supplying moisture to the dermis, exerting antioxidant effects, expanding volume in the dermis and subdermal layer, and enhancing collagen production in the dermis. HA, with the ability for each molecule to bind up to 218 water molecules, prevents skin dryness and augments volume in the dermis and subdermal layers. In 2007, Wang et al. observed fibroblast extension and collagen neogenesis under an electron microscope via skin biopsies conducted at weeks 4 and 13 after injecting cross‐linked HA filler into the forearms of 11 elderly individuals.^3^ Injected HA in the dermis absorbs moisture from the ECM, expanding the overall volume by 500–1000 times its molecular size, leading to fibroblast elongation and collagen neogenesis. The elongated fibroblasts initiate the expression of connective tissue GF, transforming GF‐beta1, and transforming GF‐beta2 GFs essential for collagen neogenesis, while also expressing tissue inhibitor of metalloproteinases (tissue inhibitor of metalloproteinases‐1, tissue inhibitor of metalloproteinases‐2, tissue inhibitor of metalloproteinases‐3) genes, thereby inhibiting collagen breakdown.

As a skin booster, non‐cross‐linked HA fillers exhibit reduced volumizing effects and shorter durations compared to cross‐linked HA. However, they diffuse well into peripheral tissues, causing fewer irregularities on the skin surface post‐procedure. Therefore, they are suitable for moisturizing thin and dry areas such as the eye area. Conversely, cross‐linked HA, due to its volumizing effects and prolonged duration, is more useful in areas other than the eye region.

HA filler products, classified as skin boosters, are poised to consolidate their market presence through continual advancements. Yet, inherent limitations persist in this procedure. Primarily, its duration of effect varies in literature but typically spans around six months following three sessions. Second, discomfort during injections remains a concern. Lastly, achieving precise delivery of HA fillers to the intended site and skin layer poses a challenge. There have been recurrent inquiries about the accuracy of delivering HA fillers to the dermis. Nevertheless, with evolving and more precise delivery methods for HA into the dermis, improved outcomes are anticipated in the future.^4^

The study of Chen et al.^5^ explored a novel hyaluronan complex's effectiveness against intrinsic skin aging, revealing its multiple mechanisms. Using immunohistochemical analysis and assays, it demonstrated the complex's ability to increase type‐I collagen expression while inhibiting matrix metalloproteinase‐1 production in human fibroblasts. The complex also showed benefits in skin equivalents by enhancing dermal‐epidermal junction protein expression. This proof‐of‐concept study suggests the hyaluronan complex possesses anti‐aging effects by influencing matrix metalloproteinase‐1 expression, promoting collagen accumulation, and enhancing dermal‐epidermal junction protein expression, opening new avenues for hyaluronan research.

In recent studies, the combination of HA with the glycerol (Belotero Revive, Merz Pharmaceuticals GmbH, Frankfurt, Germany) (Figure 1) has demonstrated significant and sustained improvement in skin hydration, elasticity, firmness and glow for up to 36 weeks.^6^, ^7^ Notably, glycerol is introduced as an additional additive in these formulations. Emphasized by Schwarz et al.,^8^ moisturizers play a crucial role in preserving skin barrier integrity and regulating moisture levels, encompassing occlusives, humectants, and emollients. Glycerol, functioning as a humectant, stands out for its remarkable water‐binding ability, augmenting skin hydration and reinforcing the resilience and protective function of mature corneocytes.^9^

**FIGURE 1:** The medical device Belotero Revive, an injectable hyaluronic acid gel manufactured by Merz Pharmaceuticals GmbH, Frankfurt, Germany, is employed in esthetic dermatology to improve skin quality. Glycerol is incorporated as an additional component.

### 2.2 Poly‐L‐lactic acid and poly‐D‐lactic acid

To maintain elasticity and anti‐aging, various procedures have historically stimulated the dermis through skin puncturing or energy‐based devices. However, recent introductions include methods that stimulate the dermis not by heat or needles but through the use of skin booster ingredients.

Polymers are now employed as skin boosters. While HA fillers are valued for their naturalness and skin‐enhancing properties, their limitation lies in their short‐term volume retention when addressing concerns like scars. Hence, there is a demand in clinical settings for a skin booster filler prioritizing lasting volume retention and ensuring safety. Sculptra, utilizing poly‐L‐lactic acid (PLLA) as an alternative material, has been employed to fulfill this need.^10^ Sculptra was initially effective in stimulating extensive collagen synthesis, particularly in patients with rapid facial volume loss like those affected by acquired immunodeficiency syndrome. However, there have been ongoing concerns related to particle irregularities, size variations, unevenness, protrusions, and the formation of granulomas. In response to these challenges, PLLA, an isomer of poly‐lactic acid, has been developed. Products such as BLLV® (Sihler Inc., Korea) have improved particle size uniformity and reduced sizes while incorporating HA instead of carboxymethylcellulose (Figure 2). Despite this improvement, the use of polymer‐based products within the dermal layer continues to evoke uncertainties among physicians, necessitating long‐term observation for potential immune reactions involving large‐scale giant cells.^11^, ^12^ This is reminiscent of the experience encountered with granulomas in the past when using PLLA. Additionally, there are skin boosters that provoke the tissue by injecting a high‐concentration solution, which involves the use of hypertonic dextrose solution. This material is commonly utilized in prolotherapy for pain management and rehabilitation therapy. According to Regina et al. in 2016, hypertonic dextrose solution is water‐soluble and is considered an ideal proliferant due to its safety even in large quantities placed in multiple areas of the body's fluid components.^13^ The cosmetic use of hypertonic dextrose has been limited to certain dermatological practices so far, and evidence supporting its esthetic use remains scarce.

**FIGURE 2:** Poly‐L‐lactic acid (PLLA), an isomer of poly‐lactic acid, has been developed. BLLV (Sihler Inc., Korea) (A) demonstrate enhanced particle size consistency and reduced sizes by utilizing hyaluronic acid instead of carboxymethylcellulose, as observed through scanning electron microscopy (B).

### 2.3 Deoxyribonucleic fragments (polydeoxyribonucleotide and polynucleotides)

Polynucleotides (PN) have gained increasing popularity in global esthetic and cosmetic applications due to their exceptional biocompatibility. Derived from chum salmon or trout gonads, PN stands out from other biostimulators as it is sourced from natural origins rather than being synthetic polymer‐based products. Significantly, PN and polydeoxyribonucleotide (PDRN) differ across several aspects: PN originates from testes, whereas PDRN is obtained from sperm cells. Notably, PN features longer nucleotide chains and a higher molecular weight, as evidenced in recent research. Moreover, PN showcases a distinct scaffold structure, setting it apart from PDRN formulations. In 2014, the first PN used as the skin booster was Rejuran® (Figure 3).

**FIGURE 3:** Rejuran (Pharmaresearch Inc., Korea) is one of the polynucleotide products used for skin rejuvenation, offering various viscosities and components, including lidocaine and hyaluronic acid.

In 1989, Bruroni et al. implemented PDRN in patients with cervical ectropion,^14^ followed by Perino et al.’s utilization of PDRN for post‐cauterization re‐epithelialization in 1990.^15^ Furthermore, Muratore et al.^16^ conducted research in 1997 involving human placental PDRN on primary cultured human knee skin fibroblasts. Subsequently, in 1999, Thellung et al. published a significant article elucidating the role of A2A receptors in PDRN's mechanism of action.^17^ Additional studies have delved into the application of PDRN in diverse areas such as skin graft donor site healing,^18^, ^19^ stimulating corneal fibroblasts in culture, promoting human osteoblast proliferation,^20^, ^21^ and facilitating angiogenesis.^22^, ^23^

One noteworthy discovery is PDRN's ability to enhance cyclobutene pyrimidine dimer repair in ultraviolet B‐exposed dermal fibroblasts.^24^ Recent research has also uncovered various properties of PDRN, including its role in antimelanogenesis,^25^, ^26^ anti‐allodynic effects,^27^ mitochondrial biogenesis,^25^ and its potential application in inducing fat browning for anti‐obesity purposes.^28^ Conversely, PNs consist of longer chains of nucleotides and have comparatively fewer research studies supporting their effects. In 2016, Park et al. demonstrated that PN improved various skin parameters such as pore size, skin thickness, tone, melanin levels, wrinkles, and sagging in a study involving five patients.^29^ Similarly, in a randomized, double‐blinded, controlled trial by Kim et al. in 2018, 44 patients who underwent thyroidectomy showed considerable improvements in post‐surgery scars when treated with PN. This improvement was evidenced by significantly enhanced Vancouver Scar Scale scores, three‐dimensional analysis of height, improved patient satisfaction, and reduced erythema index.^30^

In 2022, Lee et al. conducted a randomized, double‐blind, split‐face trial involving 27 subjects who received injections of PN and non‐cross‐linked HA filler. The study revealed that the PN group exhibited greater improvement rates in pore volume and roughness compared to the other group. However, the improvement observed did not reach statistical significance concerning global esthetic improvement scale, visual analog scale, or dermal density.^31^ In recent developments, Kim et al. published two cases demonstrating the successful use of PN in volumizing facial areas that were conventionally treated with other types of dermal fillers.^32^ Lee et al. conducted a survey involving 557 Korean physicians, revealing that a significant majority of doctors employed PN to address various facial erythema issues. More than 80% of the surveyed physicians considered PN treatment as “effective” or “highly effective.”^33^ Crucially, across the aforementioned studies, two key points stand out: First, there were no documented instances of serious adverse events, underscoring the safety profile of the treatment. Second, while the mechanism of action remains uncertain, it is postulated that owing to the molecular similarity between PN and PDRN, PN may operate through a mechanism akin to that of PDRN. However, as of now, this supposition lacks scientific substantiation.

### 2.4 Platelet‐rich plasma

Platelet‐rich plasma (PRP) is plasma with highly concentrated platelets obtained from autologous blood. Platelets in PRP contain several components such as clotting factors, GFs, chemokines, and cytokines.^34^ These components induce cellular growth and skin homeostasis, allowing PRP to benefit biological regeneration. PRP, freshly isolated from blood, exists in a noncoagulated state before activation of platelets to release GFs present within them, allowing for their beneficial utilization.

Platelets, originating from megakaryocytes, lack a nucleus, with a diameter of 2–3 μm and a thickness of approximately 1.5 μm, and have a lifespan of about 8–10 days. One‐third of the body's platelets are stored in the spleen, while the remaining two‐thirds circulate in peripheral blood. PRP has gained popularity as a prominent skin booster in cosmetic applications due to the proven efficacy showcased in various studies, primarily attributed to numerous physiological active substances contained within platelet storage granules.

Platelet storage granules include three types: alpha granules, lysosomal granules, and dense granules, among which alpha granules house a multitude of GFs.^35^

The alpha granules contain GFs such as platelet‐derived GF, transforming GF‐beta (TGF‐β), vascular endothelial GF, epithelial GF, along with von Willebrand factor, fibronectin, fibrinogen, vitronectin, clotting factors (blood clotting factors V, protein S), antifibrotic substances, chemokines, and others.

Lysosomal granules store various digestive enzymes. Dense granules contain substances like serotonin, adenosine diphosphate), adenosine triphosphate, and several glycoproteins present on the platelet membrane that play crucial roles in primary hemostasis.

PRP comprises 94% platelets, 5% red blood cells, and 1% white blood cells. To achieve clinical effectiveness, a specific platelet threshold is required in PRP. Typically, it is recommended to have at least one million platelets per microliters or 4–7 times the normal platelet count.

The core principle of PRP therapy involves activating the numerous cytokines or GFs within platelets by adding autologous thrombin or ionized calcium during the activation process of well‐concentrated PRP. These cytokines stimulate wound healing and tissue regeneration.

PRP production includes a single‐spin method and a double‐spin method based on centrifugation. Recently, the single‐spin method has gained popularity due to the availability of various user‐friendly PRP kits and one of them is the NRP20, the widely acknowledged PRP kit used in Korea, which is equipped with a centrifuge tube (N‐Finders, Korea) to facilitate the separation of these components (Figure 4).

**FIGURE 4:** The single‐spin method has gained popularity due to the availability of user‐friendly PRP kits, such as NRP20 (A), a widely acknowledged PRP kit in Korea. It is equipped with a centrifuge tube (N‐Finders, Korea) to facilitate the separation of components (B).

Facial aging shows a decreased number of fibroblasts with reduced collagen production and other ECM proteins, resulting in wrinkles, loose skin, coarseness, and pigmentation.^36^ PRP may induce ECM remodeling and stimulate fibroblast proliferation of skin and collagen synthesis thus repairing general signs of skin aging. When PRP is injected in dermis, it causes a mild inflammatory reaction of skin, stimulating the healing process. As a result, collagen synthesis is triggered, and the skin may become tightened and strengthened.^37^ Skin condition improvement is noticeable within 3 weeks. Full collagen reproduction requires approximately 3 months.^38^, ^39^ In one study, three sessions of intradermal PRP were conducted on 12 female patients. The injections are applied on the forehead, crow's feet area, cheeks, and nasolabial folds.^40^ The improvements were evaluated by patient's satisfaction questionnaire, imaging, and investigators. No serious side effects were observed. According to the imaging and satisfaction questionnaire, the result showed improved skin texture, elasticity, barrier function, and wrinkles.^40^ In a recent blinded split‐face study, the efficacy of PRP dermal injection on aged facial skin. Saline dermal injection was a control group. The mean photoaging score of 19 participants was rated by two dermatologists. Skin texture, wrinkles, pigmentation, and telangiectasis were improved on PRP injected side. However, fine lines, mottled pigmentation, roughness, and sallowness showed no significant difference.^41^ In order to evaluate the efficacy of PRP therapy for rejuvenation, Abuaf et al.^42^ performed a punch biopsy on human skin. The samples were taken from an infra‐auricular area in three different timelines, before injection, 28 days after PRP injection, and 28 days after saline injection PRP injected group showed increased collagen fiber and elastic fibers compared to control group and saline‐injected group. These effects allow PRP therapy to help improve wrinkles, hypertrophy scars, skin tones, and other inflammatory conditions. However, the efficiency of PRP skin booster does not depend on dosage difference.^43^ Five percent PRP showed more induced collagen synthesis than 10% PRP. Additionally, a greater number of fibroblast proliferation was observed in 5% PRP than 10% PRP. PRP as skin booster is usually performed by microneedling or micro‐injection and showed no significant difference in improvement between these techniques.^44^ According to many studies, PRP has relatively low risk of side effects than other skin rejuvenation treatments because it is autologous‐derived product. Possible side effects are pain, infection, redness, swelling, and bruising. Despite its simple and rapid process of PRP production thus gaining a growing popularity as a skin rejuvenation therapy, the efficacy and safety of PRP therapy remain controversial.

### 2.5 Growth factors

Throughout history, GFs have stood as one of the earliest iterations of skin boosters. Renowned for their capability to stimulate diverse cells and support the healing of wounds, these factors have been administered into the skin using techniques such as PRP. Moreover, there is a growing trend of incorporating GFs into cosmetic products as constituent known for its skin‐enhancing properties.^45^

In addition, nearly all products are formulated with components that either encompass GFs or facilitate their generation.^46^ Yet, the majority of cell receptors that receive GFs come from damaged cells rather than normal cells.^47^ It is essential to contemplate the potential advantages of providing GFs to healthy skin. The authors hypothesize that GF therapy might exhibit greater effectiveness in triggering wound healing processes when accompanied by stimuli like energy‐based devices or needling. Additionally, it requires a certain duration for diverse GF receptors to become fully established at the onset of the wound‐healing process.

Since Cohenn elucidated the role of epidermal GF (EGF) in cell division in 1986, GFs have been recognized as fundamental elements in cell regeneration. Various research findings have confirmed the requirement for diverse GFs at different stages of tissue injury healing. They have been identified as the most direct and effective factors acting upon injury. Additionally, numerous vitamins are associated with the process of skin aging. Vitamin C, for instance, accelerates DNA synthesis and acts as an essential antioxidant crucial for collagen synthesis. Vitamin A plays a significant role in regulating epidermal regeneration and melanin cell activity, exhibiting antioxidant effects that, combined with Vitamin C, aid in the synthesis of collagen and other ECM components. Vitamin E contributes to regulating skin physiological regeneration and facilitates recovery in damaged skin. Vitamin B is essential for numerous cellular functions, serving as a catalyst in the generation, breakdown, and transfer of energy from carbohydrates, fats, proteins, and the synthesis of various biomolecules.

Among minerals, calcium primarily regulates cellular homeostasis, while phosphorus is crucial for cell wall formation and other biological membranes. Furthermore, magnesium is essential for maintaining numerous normal enzyme reactions and plays a vital role in normal cell function. Amino acids promote fibroblast proliferation, stimulate collagen synthesis, generate GFs, and reduce the rate of collagen breakdown.

Usually, based on the available literature, besides PDGF, it generally requires around 12–24 h for receptors to be completely developed.^48^ Hence, it is important to assess the usefulness of employing GFs in a scenario where receptor safety might be compromised.^49^ The majority of GFs possess a positive charge, which poses a significant challenge during the skin penetration stage. However, upon reaching the dermis, where cells carry a negative charge, these factors tend to be attracted towards them. Notably, the epidermis in wounds also holds a negative charge, facilitating the penetration of GFs. Solely relying on the natural skin absorption of GFs without employing various absorption‐enhancing methods might not yield optimal results. Recently, diverse GFs have found application in skin pigment therapy. For instance, endothelial GF is recognized for its ability to inhibit melanogenesis and reduce tyrosinase activity, making it a viable option for addressing post‐laser pigmentation issues. Furthermore, understanding and discerning the utilization of different GFs are pivotal in achieving desired outcomes. An example of a skin booster that utilizes a multitude of growth factors cultured by fibroblasts (QTcell, S.THEPHARM Co., Ltd., Seoul, Korea). The skin‐booster incorporates a distinctive cultivation technique termed “Functionally Enhanced Cell Spheroid” into cultivation of human dermal fibroblasts. In this process, cells loosely adhere to the recombinant protein matrix, concurrently inducing cell to cell binding.^50^ With prolonged culture time, interactions among cells surpass those between cells and the matrix, resulting in the formation of uniform spheroids (Figure 5). This technique significantly increases the concentration of growth factors such as FGF, HGF, and PDGFRa.

**FIGURE 5:** The growth factor based skin booster produced by fibroblast (QTcell by S.THEPHARM Co., Ltd. in Seoul, Korea) (A). This skin‐booster adopts a unique cultivation method called “Functionally Enhanced Cell Spheroid” for growing human dermal fibroblasts (B). During this technique, cells loosely attach to a protein matrix, prompting simultaneous cell‐to‐cell connections.

### 2.6 Exosome

In recent years, the field of dermatology and esthetics has seen a notable surge in the application of secretome and exosome. These advancements are driven by a deepening understanding of cellular communication and regenerative medicine. They are being harnessed to deliver specific GFs, proteins, and genetic materials directly to target cells, enhancing tissue repair and regeneration. Skin boosters are a range of ingredients that improve the extracellular matrix of the dermis to enhance the skin's condition. Exosome are one of a series of skin booster products that have been widely discussed in recent years. Although further exploration and in‐depth research are still requires regarding the source of materials, efficacy, safety, and potential additional benefits, several studies have provided sufficiently good and promising explanations and results. Here is a brief explanation of the mechanism of exosome application in improving quality at each layer of the skin. Exosomes, the smallest type of extracellular vesicles, with a size range of 30–110 nm, encapsulate proteins, mRNA, miRNA, and lipids within a lipid bilayer derived from the cell membrane, contributing significantly to the stages of wound healing and skin rejuvenation. Exosome despite being plentiful in nature, present significant challenge in extraction and stabilization owing to their diminutive size and sensitivity to fluctuations in temperature, pressure and pH. Although numerous sources and techniques for isolation and stabilization have been suggested, there remains a lack of a universally accepted method for their isolation and purification.^51^ Exosomes are small extracellular vesicles secreted by cell types and are a main component of cellular communication and molecule transportation. They are responsible for extensive intercellular communication in the form of cellular components such as proteins, miRNA, nucleic acids, and various metabolites.^52^

Photoaging, a consequence of environmental factors like ultraviolet radiation and other stressors, significantly impacts skin quality. Recent medical advancements have focused on mesenchymal stem cells and noncoding RNAs, which exhibit promising potential in combating photoaging due to their ease of collection and diverse physiological roles. The study of Li et al. highlights the significant clinical promise of stem cells and their derivatives, including exosomes and noncoding RNAs, in rejuvenating aging skin and mitigating the effects of photoaging.^53^ Applying exosomes directly after skin rejuvenation treatments like fractional laser, microneedling, radiofrequency micro‐needling, and microdermabrasion aids in the healing process. This approach helps to mitigate symptoms associated with these procedures, including erythema, edema, and discomfort.^51^ Exosomes have been demonstrated to expedite the transition from inflammatory wound repair to the remodelling phase by diminishing the expression of inflammatory factors. Research indicates that mesenchymal stem cell exosomes influence macrophage polarization by targeting PKNOX1. This action leads to a reduction in the expression of inflammatory factors such as interleukin‐10 and tumor necrosis factor‐alpha, effectively managing the inflammatory response.^54^ Exosomes play a crucial role in cell communication within the epidermis, significantly affecting keratinocyte behaviour. These small extracellular vesicles facilitate the transfer of proteins, lipids, and RNA between cells, thereby influencing various cellular functions. They do so by promoting cellular cohesion and stratification which are essential for a robust and effective skin barrier.^55^ The behaviour of keratinocytes, the predominant cell type in the epidermis, is also significantly influenced by exosomes. These vesicles aid in the regulation of keratinocytes proliferation and differentiation, processes that are fundamental to maintaining the structural integrity and function of the epidermis. Through the delivery of specific molecular signals, exosomes guide these cells in responding appropriately to various environmental stimuli, thereby contributing to the skin's adaptive capacity.^56^

Exosome serve as key messengers within the dermis, significantly iinfluencing the behaviour of fibroblast, the cells chiefly responsible for the production of collagen and elastin. These two proteins are crucial for maintaining skin elasticity and strength. Exosomes facilitate the communication between skin cells and fibroblast function, enhance collagen and elastin synthesis, and increase dermal fat, thus promoting the regenerative and restorative capacity for skin anti‐aging. This results improved skin texture and a reduction in the appearance of wrinkles and fine lines. Exosomes also play a role in elastin production, this elastic property is essential for maintaining a youthful and firm skin appearance.^57^ At the molecular level, exosomes exert their rejuvenating effects through various pathways and GFs, notably TGF‐B. It plays a critical role in skin repair and rejuvenation, influencing cell growth, proliferation, and differentiation. Exosomes carry and deliver TGF‐B to target cells in the skin, thereby triggering specific signaling cascades that lead to improved skin structure and function.^57^, ^58^ Furthermore, exosomes are involved in the modulation of the ECM, a complex network of proteins and other molecules that provide structural and biochemical support to surrounding cells. They assist in the remodeling of this matrix, a process that is particularly important in wound healing and in the prevention of scar formation.^59^ Recently, there has been a growing focus on exosomes derived from the human pharynx (Exodew, Hyundaimeditech Inc, Korea). Stem cells collected through swab‐based sampling during examinations such as influenza from early childhood are known for their exceptional differentiation capabilities (Figure 6).

**FIGURE 6:** Recently, there has been a growing emphasis on exosomes derived from the human pharynx (Exodew, Hyundaimeditech Inc., Korea) (A). Stem cells collected through swab‐based sampling during examinations in pharynx (red dotted), such as influenza in early childhood, are recognized for their remarkable differentiation capabilities (B).

### 2.7 Secretomes

The secretome refers to the comprehensive collection of soluble components that a cell releases into its surrounding environment. This includes various molecules such as GFs, cytokines, and peptides, as well as insoluble particles like extracellular vesicles and exosomes. Dermal fibroblasts are known to secrete a diverse array of GFs, cytokines, and exosomes, serving as essential mediators of communication with neighboring cells to support and facilitate the maintenance and repair of the ECM. Notably, a number of products advertised as “growth factor” are actually secretome products, which consists of exosomes. Recent scientific advancements have shed light on the critical role played by extracellular vesicles, particularly exosomes, in the intricate cellular communication processes involved in various biological functions, including wound healing and skin repair.^51^, ^60^

Secretomes can be derived from various sources, including bone marrow, adipose tissue, neonatal tissue, skin tissue, and peripheral blood. They have been shown to enhance the migration and proliferation of various dermal cells, including fibroblasts, endothelial cells and keratinocytes, and the epidermis.^61^ Animal studies showed that secretomes reduce wrinkle formation, improve skin hydration, and increase collagen synthesis based on Masson‐trichrome analysis.^62^, ^63^

The ability of secretome and exosome to influence key cellular processes underscores their potential in advancing skin care and dermatological treatments. This innovative approach is revolutionizing personalized skincare treatments and noninvasive esthetic procedures, offering more effective alternatives compared to other modalities. The integration of these bio‐molecular technologies signifies a pivotal shift towards more sophisticated, targeted, and natural approaches in dermatological therapies and esthetic enhancements.

### 2.8 Chitosan

Chitosan is a polysaccharides extracted from crabs and fungi, and many studies have been conducted on various cell signaling in stem cells, platelets, and immune cells, and tissue regeneration.^64^, ^65^, ^66^

One of the chitosan's main regenerative mechanisms is to promote proliferation and differentiation of stem cells. In particular, it is known that by upregulating the expression of stromal‐derived factor‐1α, it induces the homing of stem cells and angiogenesis, thereby enhancing regeneration.^67^

Issaragrisil et al. reported that chitosan promotes the proliferation and differentiation of human mesenchymal stems, and its ability to enhance migration of stem cells was identified in vitro.^68^

Wang et al. studied the vessel formation of chitosan hydrogel and its tissue regeneration ability. They compared the effectiveness in the ischemic myocardial infarction model with adipose‐derived stem cells and showed that chitosan hydrogel induced new blood vessels and inhibited fibrosis at a similar level to adipose‐derived stem cells.^69^

Based on the biological function of chitosan materials, a study was published that applied chitosan to regenerative dermal filler. Park et al. applied liquid‐to‐gel technology to formulate a liquid chitosan material to gel in dermal tissue, and announced that this material shows high durability after being injected into the skin and promotes collagen production compared to HA filler.^70^

Medifab's Res Novae is a skin booster based on carboxymethyl chitosan with the above regenerative mechanism. They demonstrated that carboxymethyl chitosan skin booster with liquid‐to‐gel technology recruited CD29+ mesenchymal stem cells in dermal tissue (Figure 7).

**FIGURE 7:** The first Kitosan‐based skin booster, Res Novae (Medifab Inc., Korea) (A), was released, and a recent study found that Kitosan recruited CD29+ mesenchymal stem cells into the dermal tissue of SKH‐hairless mice at day 1 after intradermal injection (B). Scale bar: 100 μm. DAPI, 4′,6′‐diamidino‐2‐phenylindole; PBS, phosphate‐buffered saline.

Considering the above mechanisms, it is expected that chitosan material can be used as a new regenerative material that enhances skin tissue regeneration by activating intrinsic stem cells.

### 2.9 Botulinum toxin

The hyper‐dilution with intradermal delivery of BoNT, sometimes called “microbotox” or “babybotox,” has been shown to rejuvenate the facial skin.^71^, ^72^ Several studies have shown the benefits of using BoNT to improve facial flushing and erythema.^73^, ^74^, ^75^ The suppression of vascular endothelial GF, a major angiogenetic factor, expression by BoNT is considered as a possible mechanism.^76^ One split‐face controlled study by Sayed et al. reported the significant reduction of sebum production and pore size after BoNT intradermal injections and the results lasted long up to 4 months after treatment.^77^ Furthermore, increasing collagen production by BoNT injection has been investigated and shown the promising results.^71^ More collagen deposition seemed to be observed through Masson trichrome stain on histological examination 2 months after BoNT type A (BoNT‐A) intradermal injection in the study of Chang et al.^78^ It affects the interaction between acetylcholine and its receptors (alpha 3 nicotinic acetylcholine receptor; alpha 7 nicotinic acetylcholine receptor) in fibroblasts to regulate collagen homeostasis.^79^, ^80^

Interestingly, recent clinical studies have reported positive effects of BoNT‐A on skin pigmentation.^81^, ^82^ It is shown to terminate ultraviolet‐induced skin pigmentation by inhibiting tyrosinase activity and melanocyte activity. Jung et al. investigated the intracellular penetration of BoNT in cultured human epidermal melanocytes, and human epidermal keratinocytes. The study revealed that melanocytes and keratinocytes exhibited uptake of BoNT and showed the ability to inhibit epidermal melanin production.^83^

In terms of clinical application, BoNT should be delivered intradermally, uniform‐sized, droplets for the effective outcomes. The hyper‐dilution with minimal dosage is used for this condition. However, if dosage is too little, it will create an inadequate result, while, too high dosage might create undesirable outcome due to unintentional effect to deeper facial muscle fibers. The injection technique requires the use of a 30‐ or 32‐G needle, creating a small wheal of the product with 0.03–0.05 mL in numerous small droplets per point at 0.8–1.0‐cm intervals in a grid‐like pattern. The duration of the effect generally maintains for 1–3 months. Moreover, the more advantageous usage of BoNT for skin rejuvenation is that it can be mixed with other injectables called “mesococktails” to optimize treatment outcome without losing the efficacy of each product.^84^ BoNT can provide promising outcomes in order to improve skin quality and facial rejuvenation. Several aspects of good skin quality can be achieved by BoNT‐A intradermal administration. It offers cost‐effectiveness, minimal side effects, and sensible duration of action. Moreover, it can integrate with other modalities as well as the ability to create combination injectables to enhance treatment outcomes. Unsurprisingly, BoNT‐A is widely embraced in the several esthetic indications.

## 3 DISCUSSION

A critical factor in optimizing the efficacy of skin boosters involves effectively delivering the active components through the skin's protective barrier. The challenge lies in finding methods that facilitate ingredient penetration into the dermal layers without causing discomfort.

Several approaches can be employed to achieve this, including injection techniques like mesotherapy, iontophoresis, electrophoresis, microneedling, high‐frequency needling, ultrasound, laser, plasma, and transcutaneous drug delivery using needleless injectors. The chosen delivery method is just as pivotal as the selection of the skin booster itself.^85^, ^86^

For instance, previously, the subcutaneous injection of PDLA, a type of polymer, was typically administered via needle injection. However, with the advancement of microinvasive needling techniques, subcutaneous injections are now achievable through machine‐based control methods.

When injecting skin boosters into the skin, the process often involves the use of needles or the application of mechanical pressure to deliver the injection into the tissue. The effects stemming from these procedural steps should be duly considered. Studies on the impact of needle‐induced skin tissue stimulation have elucidated the effects of mechanical stimulation on fibroblast cells. For instance, Langevin's research highlighted the influence of needles on local tissues and their effects on fibroblast cells (Figure 8).^87^ It was noted that external forces on cells can lead to cell shrinkage, thereby exerting stress on fibroblasts, affecting various cellular metabolisms. Additionally, experiments conducted by Langevin in 2006^88^ demonstrated an increase in fibroblast cell activity when the needle, after penetrating subcutaneous tissue, was twisted experimentally (Figures 9 and 10). This illustrates how mechanical stimulation alone can potentially regulate fibroblast cell activity in clinical settings. Such findings can be applicable not only to procedures involving needle penetration of the skin but also to various other interventions utilizing injectable substances.

**FIGURE 8:** Studies on the impact of needle‐induced skin tissue stimulation have elucidated the effects of mechanical stimulation on fibroblast cells. For example, Langevin's research highlighted the influence of needles on local tissues and their effects on fibroblast cells. FB, Fibroblast cell, FB.

**FIGURE 9:** Langevin's experiments demonstrated an increase in fibroblast cell activity when the needle, after penetrating subcutaneous tissue, was experimentally twisted.

**FIGURE 10:** Through mechanotransduction, cells receive signals to the cytoplasm and cell nucleus through the deformation of the cell wall. This process sends signals to the cell nucleus for cell differentiation, division, growth, protein synthesis, and initiates the remodeling of the cellular cytoskeleton.

In conclusion, the term “skin booster” has not previously had a defined scope, but it broadly encompasses all substances that, when injected or applied to penetrate the dermis, influence skin rejuvenation.

## CONFLICT OF INTEREST STATEMENT

I acknowledge that I have considered the conflict of interest statement included in the “Author Guidelines.” I hereby certify that, to the best of my knowledge, no aspect of my current personal or professional situation might reasonably be expected to significantly affect my views on the subject I am presenting.

## ETHICS STATEMENT

All analyses are based on previously published data and studies. This article adheres to ethical standards in scholarly writing and citation. No confidential or personal data have been used, and all sources have been appropriately credited to respect intellectual property rights and academic integrity. The content presented in this review is solely for educational and informational purposes and does not require ethical approval as per institutional guidelines.

## Data Availability

The data that support the findings of this study are available from the corresponding author upon reasonable request.
